# Smoking can increase nasopharyngeal carcinoma risk by repeatedly reactivating Epstein‐Barr Virus: An analysis of a prospective study in southern China

**DOI:** 10.1002/cam4.2083

**Published:** 2019-03-07

**Authors:** Ting Hu, Chu‐Yang Lin, Shang‐Hang Xie, Geng‐Hang Chen, Yu‐Qiang Lu, Wei Ling, Qi‐Hong Huang, Qing Liu, Su‐Mei Cao

**Affiliations:** ^1^ Department of Cancer Prevention State Key Laboratory of Oncology in Southern China Collaborative Innovation Center for Cancer Medicine Guangdong Key Laboratory of Nasopharyngeal Carcinoma Diagnosis and Therapy Sun Yat‐sen University Cancer Center Guangzhou People's Republic of China; ^2^ School of Public Health Sun Yat‐sen University Guangzhou People's Republic of China; ^3^ Sihui Cancer Institute Sihui People's Republic of China

**Keywords:** Epstein‐Barr Virus, nasopharyngeal carcinoma, reactivation, smoking

## Abstract

**Background:**

The association between smoking and nasopharyngeal carcinoma (NPC) is still uncertain. The aim of this study was to validate smoking effect on NPC and explore if smoking can induce NPC by persistently reactivating EBV in long‐term based on a prospective cohort design.

**Methods:**

A NPC screening cohort with 10 181 eligible residents in Sihui city, southern China was conducted from 2008 to 2015. The smoking habit was investigated through the trained interviewers and EBV antibodies (VCA‐IgA, EBNA1‐IgA) as screening markers were tested periodically. New NPC cases were identified through local cancer registry. Cox's regression model was used to estimate the adjusted hazard ratios (aHRs) of smoking on NPC incidence. In the non‐NPC participants, the associations between smoking and EBV seropositivity in different periods were assessed by logistic regression and generalized estimating equations (GEE).

**Results:**

With a median of 7.54 years, 71 NPCs were diagnosed ≥1 year after recruitment. Compared with never smokers, the aHRs of developing NPC among ever smokers were 3.00 (95%CI: 1.46‐6.16). Stratified by sex, the HRs of ever smoking were 2.59 (95%CI: 1.07‐6.23) for male and 3.75 (95%CI: 1.25‐11.20) for female, respectively. Among the non‐NPC individuals, ever smoking was not only associated with EBV seropositivity at baseline, but also in the 3‐5 years of follow up, with adjusted odds ratios (aORs) of 1.68 (95%CI: 1.29‐2.18) for VCA‐IgA and 1.92 (95%CI: 1.42‐2.59) for EBNA1‐IgA. Among the smokers who were tested EBV antibodies at least twice, the similar results were obtained using GEE.

**Conclusion:**

Smoking could significantly increase the long‐term risk of NPC in southern China, partly by persistently reactivating EBV.

## 1 INTRODUCTION

Nasopharyngeal carcinoma (NPC) is rare in most populations around the world, with an incidence of usually less than one per 100 000 person‐years. However, this malignancy is prevalent in most of Southeast Asia and southern China with incidence rates of 5‐20 and 20‐50 per 100 000 person‐years, respectively.^1^, ^2^, ^3^ Epstein‐Barr Virus (EBV) is considered a necessary etiologic factor of NPC in endemic areas.^4^, ^5^, ^6^ Virus DNA is consistently detected in all NPC tissues and some EBV genes have been shown to induce the transformation of premalignant nasopharyngeal epithelial cells.^7^, ^8^ EBV's transition from the latent to lytic phase is suggested as a key step in the development of NPC. Generally, EBV preferentially infects within memory B cells in latency from Waldeyer's ring and then colonizes the entire peripheral lymphoid system by trafficking with memory B cells as they circulate through the body and back to Waldeyer's ring.^9^, ^10^ Spontaneous lytic reaction of EBV is normally induced by the cellular factors, such as X‐box‐binding protein 1 (XBP‐1)^11^ or B‐lymphocyte‐induced maturation protein 1 (BLIMP1), during the differentiation of B cells into plasma cells or in the more differentiated epithelial cells.^12^ Once the lytic EBV invades mucosal tissues, the mucosal B cells are activated in regional mucosa‐associated lymphoid tissue and switched to effector cells to secrete immunoglobulin A (IgA) antibodies, which response to local presence of virus‐encoded neoantigens, to against the virus.^13^, ^14^

In healthy individuals, the virus can be periodically activated by endogenous and environmental stress factors, including hormones and cytokines,^15^, ^16^, ^17^ and food components such as butyrates and nitrosamines,^18^ which all have been shown to reactivate EBV from latency and contribute to risk of malignancy. Such virus reactivation is reflected by increased and aberrant antibody responses against multiple EBV antigens.^19^, ^20^ Several prospective epidemiological studies are convinced that EBV antibodies can be elevated for several years prior to NPC diagnosis.^21^, ^22^, ^23^ Specific antibodies, immunoglobulin A (IgA) antibodies against EBV capsid antigens (VCA‐IgA), and nuclear antigen1 (EBNA1‐IgA) have been used to screen for NPC in endemic areas. However, the fact that approximately 95% of the world's population sustains asymptomatic EBV infection with relatively low NPC incidence suggests the involvement of other genetic or environmental cofactors in the etiology of NPC.^5^, ^24^, ^25^

Smoking has been suggested as a moderate risk factor of NPC for decades. In a recent meta‐analysis, the pooled estimated Odds Ratio of smoking for developing NPC in 27 case‐control studies was 1.61 (95% CI: 1.36‐1.91),^26^ whereas four cohort studies presented a null association with OR = 1.11 (95% CI: 0.84‐1.48). Tobacco is a complex mixture that contains >4000 compounds, many of which could act as mutagens and DNA‐damaging agents that drive tumor initiation in the nasopharynx.^27^ Besides, it was hypothesized that cigarette smoking might modulate the reactivation of EBV, further inducing carcinogenesis of the nasopharynx. Several cross‐sectional studies have indicated that cigarette smoking was associated with EBV seropositivity.^28^, ^29^ Laboratory evidence also supports this viewpoint, an in vitro experiment found that exposure to nicotine promoted NPC cell proliferation and EBV replication with expression of its lytic gene products.^30^ However, few prospective large‐scale studies have evaluated the long‐term influence of smoking on EBV reactivation status.

In this study, we evaluated the effect of cigarette smoking on NPC incidence based on a prospective screening program in southern China and explored the relationship between smoking and EBV reactivation in different periods in healthy participants.

## 2 MATERIALS AND METHODS

### 2.1 Study population recruitment

Eligible participants were recruited in an NPC screening project from 2008 to 2015 in Sihui county, Guangdong province, southern China.^31^ In brief, local residents aged between 30 and 69 years old were recruited from seven towns in Sihui and invited to donate 6 mL of blood and complete a life and environmental interview questionnaire. Two EBV serologic antibodies (VCA‐IgA and EBNA1‐IgA) were used as screening markers. The participants were divided into high‐risk, medium‐risk, and low‐risk subgroups by using a defined prediction formula combined with these two markers.^32^ High‐risk individuals were referred for a nasopharyngeal fiberscope examination, and a biopsy was taken if suspicious lesions were found. Screening tests were repeatedly conducted according to the screening protocol. The high‐risk and medium‐risk individuals were retested every 1‐2 years, while the follow‐up interval for low‐risk individuals was 4‐5 years. Informed consents were obtained from all participants. This research project was approved by the Institutional Research Ethics Committee of Sun Yat‐sen University Cancer Center.

A total of 10 839 residents participated in the NPC screening cohort and completed the baseline survey. We excluded 630 ineligible individuals at baseline: 143 due to age, 28 participants because they had been diagnosed with NPC before recruitment, and 459 were missing important baseline information. After finishing the follow‐ups, we excluded 20 NPC cases who were diagnosed within 1 year after recruitment, as well as eight healthy participants who were followed up less than 1 year. Therefore, there were 10 181 subjects applicable for statistical analyses.

### 2.2 Interview questionnaire

Basic information was collected through face‐to‐face interviews by trained interviewers at baseline, including sex, age, education level, family history of NPC, intake of salted food, herb tea, slow cooked soup, and smoking status. Smoking was defined as having smoked at least one cigarette every 1‐3 days during a 6‐month period. Former smokers were defined as smokers who had quit smoking more than 1 year before the interview, current smokers were defined as smokers who had never given up smoking or quit for less than 1 year. Both former smokers and current smokers were collectively called ever smokers.^26^, ^28^ The information on smoking was only collected at baseline.

### 2.3 EBV serological test

The blood samples collected at baseline and follow up were divided into serum, plasma, and buffer coat after centrifugation at Sihui cancer institute. The samples were taken to the central laboratory at Sun Yat‐sen University Cancer Center (SYSUCC) through cold‐chain transportation within 6 hours and then stored at −80°C before testing. Following the manufactures’ instructions, the two screening markers VCA‐IgA (EUROIMMUNAG, Lübeck, Germany) and EBNA1‐IgA (Zhongshan Bio‐Tech Company, Zhongshan, China) were measured using the commercial enzyme‐linked immunosorbent assay (ELISA) kits.^31^, ^33^, ^34^ Levels of EBV antibodies were standardized by calculating a ratio of the optical density (OD) of the sample over that of a reference control (rOD). According to the ELISA kits’ standards, the positive criteria were ≥0.7 for EBNA1‐IgA and ≥0.8 for VCA‐IgA. To ensure the reliability of the serological results, we used a pooled serological sample as our control sample. The coefficient of variations of the assay from 2008 to 2015 for VCA‐IgA and EBNA1‐IgA was both approximately equaled 8%.

### 2.4 Follow up

New NPC cases were identified before the end of 2016 by both periodic check‐ups in screening and cancer registry at the Sihui Institute where an online cancer report was established in 1978.^1^, ^35^ To ensure the completeness of the cancer reports, Causes of Death Register provided by the local Disease Control (CDC) was also reviewed. Among the 91 NPC cases, 20 were detected within the first year and 71 were diagnosed ≥1 year after recruitment. Follow‐up durations were calculated from the recruitment day to the date of NPC diagnosis, date of death, date of loss to follow up, or the study deadline of 31 December 2016, whichever came first.

Among the participants free from NPC, 2737 retested in 3‐5 years; 1474 individuals were retested twice or more in the first 5 years. The detailed flow chart was presented in Figure 1.

**Figure 1:** Flow chart for participants from a nasopharyngeal carcinoma screening cohort study in Sihui city, Guangdong province, southern China. NPC, nasopharyngeal carcinoma; EBV, Epstein‐Barr Virus. This figure showed the population flow chart during participating the NPC screening program, including how long they were followed up, how many new NPC cases were diagnosed, and how many subjects completed antibodies test for once, twice and three times, respectively

### 2.5 Statistical analysis

Continuous variables were translated into categorical variables. Age was divided into four categories, VCA‐IgA, and EBNA1‐IgA levels were converted as positive or negative according to the above‐mentioned criteria. We defined the combined EBV antibodies as negative if both VCA‐IgA and EBNA1‐IgA were negative, else defined as positive if anyone of them was positive.

The NPC incidence rate was calculated by the number of new patients divided by the total person‐years of follow up. Cox's proportional hazard regression models were conducted to validate whether smoking influences NPC development after adjusting for sex, age, education level, family history of NPC, combined levels of VCA‐IgA and EBNA1‐IgA, alcohol use, and diet. Cox regression analyses were also carried out between different smoking status stratified by EBV antibodies’ positivity and sex. Interactions between smoking and EBV status, smoking and sex were calculated at the same time.

Among healthy individuals, odds ratios (ORs) and 95% confidence intervals (95%CIs) were calculated by logistic regression analyses to explore the influence of smoking on EBV reactivation during different follow‐up intervals (baseline and the 3‐5 years of follow up). As for non‐NPC individuals who were retested for EBV antibodies at least twice in 5 years of follow up, generalized estimating equations (GEE) were conducted to assess the association between smoking and EBV reactivation after adjusting other variables.

All data were recorded using Epidata3.1 by double entry. SAS software (version9.2, SAS institute Inc.) and SPSS19.0 (IBM Corp, Chicago, IL, USA) were used to analyze the data. All statistic tests were two‐sided with α value at 0.05.

## 3 RESULTS

After a median of 7.54 years follow‐up, 71 new NPC cases were detected ≥1 year after recruitment in this cohort, where 47 were detected by biopsy as screening process, 23 were confirmed by cancer register, and only one was certificated by causes of death register with the percentage of death certificate case as 1.4% (1/71). Among the NPCs, 26 were detected in 1‐2 years of follow up and 15 in 2‐3 years, respectively. The overall NPC incidence was 112.10 per 100 000 person‐years, with 177.63 per 100 000 person‐years for males and 65.09 per 100 000 person‐years for females, respectively.

Table 1 showed the baseline characteristics for the participants in this cohort and hazard ratios (HRs) of the risk factors associated with NPC incidence calculated by Cox regression including salted food, herbal tea, slow cooked soup, and smoking. VCA‐IgA and EBNA1‐IgA were measured for all participants at baseline, and the positive rate for combined EBV antibodies was 48.18%. Compared with the EBV seronegative groups, we confirmed EBV seropositivity was a strong risk indicator for NPC development, the adjusted Hazard Ratios (aHRs) were 5.54 (95%CI: 2.83‐10.86). Meanwhile, participants with NPC family history and frequent salted food consumption had higher risk of NPC occurrence, with aHRs of 3.43 (95%CI: 1.63‐7.23) and 2.17 (95%CI: 1.26‐3.74), respectively, confirming previous data with OR range 2‐4 for various salted food consumption.^36^, ^37^

**Table 1:** Hazard ratios (HRs) and 95% confidence intervals (CIs) of developing nasopharyngeal carcinoma (NPC) associated with smoking and other risk factors (N = 10 181) in a prospective cohort in Sihui, southern China

Variables	Participants, n (%)	Person ‐years	NPC				*P* value^b^
			Case, n	Incidence rate^a^	HR (95%CI)	Adjusted HR (95%CI)^b^	
Sex							
Male	4279 (42.03)	26 458.75	47	177.63	Reference	Reference	0.759
Female	5902 (57.97)	36 874.78	24	65.09	0.37 (0.23, 0.61)	0.89 (0.43, 1.87)	
Age, y							
30‐39	1694 (16.64)	10 199.60	17	166.67	Reference	Reference	
40‐49	3832 (37.64)	25 011.96	19	75.96	0.49 (0.25, 0.95)	0.50 (0.26, 0.99)	0.047*
50‐59	3291 (32.32)	21 321.14	26	121.94	0.76 (0.41, 1.41)	0.69 (0.36, 1.32)	0.261
60‐69	1364 (13.40)	6800.83	9	132.34	0.82 (0.37, 1.86)	0.67 (0.28, 1.58)	0.358
Education year							
<6	3883 (38.14)	24 825.68	26	104.73	0.92 (0.57, 1.49)	1.10 (0.65, 1.87)	0.718
≥6	6298 (61.86)	38 507.85	45	116.86	Reference	Reference	
Family history of NPC							
No	9841 (96.66)	61 186.05	63	102.96	Reference	Reference	0.001**
Yes	340 (3.34)	2147.49	8	372.53	3.85 (1.84, 8.04)	3.43 (1.63, 7.23)	
Combined EBV antibodies^c^							
Both negative	5276 (51.82)	32 796.77	10	30.49	Reference	Reference	<0.001**
Any positive	4905 (48.18)	30 536.77	61	199.76	6.66 (3.41, 12.99)	5.54 (2.83, 10.86)	
Smoking status							
Never smoker	7044 (69.19)	43 699.62	26	59.50	Reference	Reference	0.003**
Ever smoker	3137 (30.81)	19 633.92	45	229.20	3.84 (2.37, 6.22)	3.00 (1.46, 6.16)	
Salted food							
Less than monthly	9019 (88.59)	54 723.16	53	96.85	Reference	Reference	0.005**
Monthly and more	1162 (11.41)	8610.37	18	209.05	2.25 (1.31, 3.85)	2.17 (1.26, 3.74)	

HR, Hazard ratio; CI, Confidence Interval; NPC, nasopharyngeal carcinoma; VCA‐IgA, immunoglobulin A antibodies against EBV capsid antigens; EBNA1‐IgA, immunoglobulin A antibodies against EBV nuclear antigen1.

a Per 100 000 person‐years; *P < 0.05; **P < 0.01.

b Taking sex, age, education level, family history of NPC, EBV antibodies, smoking, salted food, herb tea, and slow cooked soup into the Cox regression model.

c Both negative: VCA‐IgA(−)/EBNA1‐IgA(−). Any positive: VCA‐IgA(−)/EBNA1‐IgA(+), VCA‐IgA(+)/EBNA1‐IgA(−), or VCA‐IgA(+)/EBNA1‐IgA(+).

NPC incidence rates among never smokers and ever smokers were 59.50 per 100 000 person‐years and 229.20 per 100 000 person‐years, respectively. The results demonstrated that smoking could substantially increase the risk of NPC incidence, with aHR of 3.00 (95%CI: 1.46‐6.16) for ever smokers. Due to much different rate for smoking among male (68.64%) and female (3.39%), we conducted Cox regression analyses stratified by sex (Figure 2). Compared with never smokers, the aHRs of ever smokers were 2.59 (95%CI: 1.07‐6.23) in male (Figure 2A) and 3.75 (95%CI: 1.25‐11.20) in female (Figure 2B).

**Figure 2:** Hazard ratios (HRs) and 95% confidence intervals (CIs) of developing nasopharyngeal carcinoma (NPC) associated with smoking and other risk factors stratified by sex (A: male; B: female). Combined EBV antibodies: Both negative indicated VCA‐IgA(−)/EBNA1‐IgA(−); Any positive indicated VCA‐IgA (−)/EBNA1‐IgA (+), VCA‐IgA (+)/EBNA1‐IgA (−), or VCA‐IgA (+)/EBNA1‐IgA (+). Abbreviations: NPC, nasopharyngeal carcinoma; EBV, Epstein‐Barr Virus; VCA‐IgA, immunoglobulin A antibodies against EBV capsid antigens; EBNA1‐IgA, immunoglobulin A antibodies against EBV nuclear antigen1. This figure included two figures (A and B). (A) displayed the number of participants, new NPC cases in each group, and showed the adjusted HRs and 95%CIs of developing NPC associated with risk factors calculated by Cox regression among male, and (B) showed the results among female

Using stratification analysis, the modified risks of NPC were calculated with the combination of smoking and EBV antibodies status, smoking, and sex (Table 2). The aHR was the greatest among the ever smokers in terms of EBV seropositivity (aHR = 12.80, 95%CI: 4.71‐34.81) compared with never smokers whose EBV was seronegative as reference. However, there was no statistically significant interaction between EBV antibody positivity and smoking status (*P *>* *0.05).

**Table 2:** The modified hazard ratios (HRs) and 95% confidence intervals (CIs) of developing nasopharyngeal carcinoma (NPC) with smoking stratified by EBV antibodies and sex in a prospective cohort in Sihui, southern China

Smoking	Variables	Participants, n (%)	Person‐years	NPC			
				Cases, n	Incidence rate^a^	HR (95%CI)	Adjusted HR (95%CI)^b^
Smoking status	Combined EBV antibodies^c^						
Never smoker	Both negative	3817 (37.49)	23 615.32	6	25.41	Reference	Reference
Never smoker	Any positive	3227 (31.70)	20 084.30	20	99.58	4.07 (1.63, 10.13)	3.80 (1.52, 9.47)
Ever smoker	Both negative	1459 (14.33)	9181.45	4	43.57	1.77 (0.50, 6.26)	1.60 (0.41, 6.28)
Ever smoker	Any positive	1678 (16.48)	10 452.47	41	392.25	15.45 (6.56, 36.41)	12.80 (4.71, 34.81)
The interaction deducting main effect of smoking and EBV: 2.11 (0.53, 8.35), *P* = 0.287							
Smoking status	Sex						
Never smoker	Male	1342 (13.18)	8158.15	6	73.55	Reference	Reference
Never smoker	Female	5702 (56.01)	35 541.47	20	56.27	0.78 (0.31, 1.95)	0.77 (0.30, 1.95)
Ever smoker	Male	2937 (28.85)	18 300.60	41	224.04	3.07 (1.30, 7.25)	2.63 (1.10, 6.28)
Ever smoker	Female	202 (1.96)	1333.32	4	300.00	4.39 (1.24, 15.59)	2.83 (0.78, 10.25)
The interaction deducting main effect of smoking and sex: 1.40 (0.35, 5.56), *P* = 0.633							

EBV, Epstein‐Barr virus; HR, Hazard ratio; CI, confidence interval; NPC, nasopharyngeal carcinoma; VCA‐IgA, immunoglobulin A antibodies against EBV capsid antigens; EBNA1‐IgA, immunoglobulin A antibodies against EBV nuclear antigen1.

a Per 100 000 person‐years.

b Adjusted for sex, age, education level, family history of NPC, EBV antibodies, salted food, herb tea, and slow cooked soup in the Cox regression model.

c Both negative: VCA‐IgA(−)/EBNA1‐IgA(−). Any positive: VCA‐IgA(−)/EBNA1‐IgA(+), VCA‐IgA(+)/EBNA1‐IgA(−), or VCA‐IgA(+)/EBNA1‐IgA(+).

We also conducted Cox regression stratified by combination of smoking status and sex. Compared with never smokers in male, the aHRs were 2.63 (95%CI: 1.10‐6.28) for ever smoker in male, and 2.83 (95%CI: 0.78‐10.25) for ever smokers in female, respectively. The interaction between smoking and sex was also insignificant.

To evaluate the long‐term effect of smoking on EBV reactivation, the associations between smoking and EBV seropositivity at baseline and the 3‐5 years of follow up were firstly calculated in non‐NPC individuals using logistic models (Table 3). With univariate analysis, the results showed smoking was associated with a higher risk of EBV seropositivity both at the baseline and 3‐5 years of follow up, with odds ratio (OR) = 1.36 (95%CI: 1.24‐1.49) for VCA‐IgA and OR = 1.34 (95%CI: 1.22‐1.47) for EBNA1‐IgA at baseline; OR = 1.29 (95%CI: 1.09‐1.52) for VCA‐IgA and OR = 1.82 (95%CI: 1.50‐2.21) for EBNA1‐IgA in the 3‐5 years of follow up. After adjusting for sex, age, education level, family history of NPC, salted food, herb tea, and slow cooked soup in the multivariable models, smoking showed similar positive associations with EBV seropositivity, with aOR = 1.40 (95%CI: 1.22‐1.60) for VCA‐IgA and aOR = 1.58 (95%CI: 1.38‐1.82) for EBNA1‐IgA at baseline; aOR = 1.68 (95%CI: 1.29‐2.18) for VCA‐IgA and aOR = 1.92 (95%CI: 1.42‐2.59) for EBNA1‐IgA in the 3‐5 years of follow up.

**Table 3:** Odds ratios (ORs) and 95% confidence intervals (CIs) of EBV seropositivity associated with smoking category in the non‐NPC individuals at baseline and the 3‐5 years of follow up

Variables	Total	VCA‐IgA (rOD ≥ 0.8)			EBNA1‐IgA (rOD ≥ 0.7)		
		N (%)^b^	OR (95% CI)	Adjusted OR (95% CI)^a^	N (%)^b^	OR (95% CI)	Adjusted OR (95% CI)^a^
Baseline							
Cigarette smoking							
Never smoker	7018	1878 (26.76)	Reference	Reference	1976 (28.16)	Reference	Reference
Ever smoker	3092	1027 (33.21)	1.36 (1.24, 1.49)	1.40 (1.22, 1.60)	1066 (34.41)	1.34 (1.22, 1.47)	1.58 (1.38, 1.82)
Smoking status							
Never smoker	7018	1878 (26.76)	Reference	Reference	1976 (28.16)	Reference	Reference
Former smoker	469	152 (32.41)	1.31 (1.07, 1.60)	1.29 (1.04, 1.60)	160 (34.12)	1.32 (1.08, 1.61)	1.52 (1.22, 1.89)
Current smoker	2623	875 (33.36)	1.37 (1.24, 1.51)	1.38 (1.20, 1.59)	904 (34.46)	1.34 (1.22, 1.48)	1.59 (1.37, 1.83)
3‐5 years of follow‐up							
Cigarette smoking							
Never smoker	1858	633 (34.07)	Reference	Reference	312 (16.79)	Reference	Reference
Ever smoker	879	351 (39.93)	1.29 (1.09, 1.52)	1.68 (1.29, 2.18)	236 (26.85)	1.82 (1.50, 2.21)	1.92 (1.42, 2.59)
Smoking status							
Never smoker	1858	633 (34.07)	Reference	Reference	312 (16.79)	Reference	Reference
Former smoker	122	52 (42.62)	1.44 (0.99, 2.08)	1.75 (1.16, 2.65)	30 (24.59)	1.62 (1.05, 2.48)	1.67 (1.04, 2.69)
Current smoker	757	299 (39.50)	1.26 (1.06, 1.50)	1.66 (1.27, 2.17)	206 (27.21)	1.85 (1.52, 2.27)	1.98 (1.44, 2.71)

NPC, nasopharyngeal carcinoma; EBV, Epstein‐Barr virus; OR, Odds ratio; CI, confidence interval; VCA‐IgA, immunoglobulin A antibodies against EBV capsid antigens; EBNA1‐IgA, immunoglobulin A antibodies against EBV nuclear antigen1; rOD, ratio of Optical Density.

a Adjusted for sex, age, education level, family history of NPC, salted food, herb tea, and slow cooked soup in logistic regression model.

b N, Participants number with positive VCA‐IgA or EBNA1‐IgA; %, Positive percentage of VCA‐IgA or EBNA1‐IgA.

At baseline, former smokers presented similar risks of EBV seropositivity with current smokers, with aOR = 1.29 (95%CI: 1.04‐1.60) vs aOR = 1.38 (95%CI: 1.20‐1.59) for VCA‐IgA and aOR = 1.52 (95%CI: 1.22‐1.89) vs aOR = 1.59 (95%CI: 1.37‐1.83) for EBNA1‐IgA. The situation was same in the 3‐5 years of follow up. The aORs of current smokers were 1.66 (95%CI: 1.27‐2.17) for VCA‐IgA and 1.98 (95%CI: 1.44‐2.71) for EBNA1‐IgA. As for former smokers, the aORs were 1.75 (95%CI: 1.16‐2.65) for VCA‐IgA, and 1.67 (95%CI: 1.04‐2.69) for EBNA1‐IgA.

For the non‐NPC individuals with repeated testing for EBV antibodies more than twice in the first 5‐year follow‐ups, we further evaluated the effect of smoking on EBV seropositivity with generalized estimating equations (Table 4). The results indicated that the risk of EBV seropositivity among ever smokers was 1.62 times (95%CI: 1.28‐2.06) for VCA‐IgA and 1.77 times (95%CI: 1.39‐2.25) for EBNA1‐IgA than never smokers. The aORs of current smokers and former smokers for VCA‐IgA positivity were 1.68 (95%CI: 1.30‐2.16) and 1.47 (95%CI: 1.04‐2.06). As for EBNA1‐IgA, current smokers showed a higher risk of seropositivity with an aOR = 1.90 (95%CI: 1.47‐2.46), and the aOR among former smokers was 1.42 (95%CI: 0.97‐2.07). There was no significant association between other factors including sex, family history of NPC, and salted food consumption. However, compared with the youngest participants, those aged 60‐69 years old were at a higher risk of EBNA1‐IgA positive status, with an aOR of 1.67 (95%CI: 1.19‐2.34).

**Table 4:** Odds ratios (ORs) and 95% confidence intervals (CIs) for EBV seropositivity associated with smoking and other factors in the non‐NPC individuals by generalized estimating equations (GEE)

Variables	N (%)	VCA‐IgA (rOD ≥ 0.8)		EBNA1‐IgA (rOD ≥ 0.7)	
		OR (95%CI)	Adjusted OR (95%CI)^a^	OR (95%CI)	Adjusted OR (95%CI)^a^
Sex					
Male	636 (43.15)	Reference	Reference	Reference	Reference
Female	838 (56.85)	0.73 (0.63, 0.84)	1.10 (0.87, 1.38)	0.79 (0.68, 0.93)	1.27 (1.00, 1.60)
Age, y					
30‐39	222 (15.06)	Reference	Reference	Reference	Reference
40‐49	628 (42.61)	0.83 (0.66, 1.04)	0.84 (0.67, 1.06)	1.03 (0.81, 1.30)	1.02 (0.81, 1.30)
50‐59	493 (33.45)	1.25 (0.99, 1.58)	1.25 (0.98, 1.58)	1.32 (1.03, 1.69)	1.30 (1.02, 1.67)
60‐69	131 (8.88)	1.38 (1.02, 1.88)	1.46 (1.07, 2.00)	1.58 (1.14, 2.18)	1.67 (1.19, 2.34)
Education year					
<6	521 (35.35)	0.87 (0.75, 1.02)	0.83 (0.71, 0.98)	0.88 (0.75, 1.04)	0.83 (0.69, 0.98)
≥6	953 (64.65)	Reference	Reference	Reference	Reference
Family history of NPC					
No	1399 (94.91)	Reference	Reference	Reference	Reference
Yes	75 (5.09)	0.95 (0.69, 1.31)	0.91 (0.67, 1.25)	0.74 (0.49, 1.11)	0.72 (0.48, 1.09)
Smoking status					
Never smoker	964 (65.40)	Reference	Reference	Reference	Reference
Ever smoker	510 (34.60)	1.63 (1.40, 1.90)	1.62 (1.28, 2.06)	1.58 (1.34, 1.85)	1.77 (1.39, 2.25)
Former smoker	87 (5.90)	1.48 (1.09, 2.03)	1.47 (1.04, 2.06)	1.28 (0.90, 1.82)	1.42 (0.97, 2.07)
Current smoker	423 (28.70)	1.66 (1.42, 1.96)	1.68 (1.30, 2.16)	1.64 (1.39, 1.95)	1.90 (1.47, 2.46)
Salted food					
Less than monthly	1256 (85.21)	Reference	Reference	Reference	Reference
Monthly and more	218 (14.79)	1.03 (0.83, 1.27)	1.06 (0.85, 1.30)	1.13 (0.92, 1.39)	1.15 (0.94, 1.42)

NPC, nasopharyngeal carcinoma; EBV, Epstein‐Barr virus; OR, Odds ratio; CI, confidence interval; VCA‐IgA, immunoglobulin A antibodies against EBV capsid antigens; EBNA1‐IgA, immunoglobulin A antibodies against EBV nuclear antigen1; rOD, ratio of Optical Density.

a Taking sex, age, family history of NPC, smoking status, salted food, herb tea, and slow cooked soup into the GEE model.

## 4 DISCUSSION

With a large‐scale cohort, our results prospectively validate smoking plays a key role in NPC development in the endemic areas of southern China, which are consistent with previous case‐control studies.^38^, ^39^ The association is independent of a handful of potential confounders, including age, sex, education level, family history of NPC, EBV infection, and dietary factors. We also confirm previous findings that family history of NPC and EBV seropositivity are both strong risk factors for NPC.^40^, ^41^

The aHR of 3.00 (95%CI: 1.46‐6.16) for NPC among ever smokers in our study was higher than the risk in another two prospective studies conducted in Taiwan 42 with aHR of 1.20 (95%CI: 0.60‐2.60) and Singapore 43 with RR of 1.10 (95%CI: 0.81‐1.49). It suggested that the residences in southern China might be more susceptive for the carcinogens in tobacco than these two high‐risk areas. In addition, our result showed that female had higher NPC risk than male when exposure to tobacco, with aHR of 3.75 (95%CI: 1.25‐11.20) in female and 2.59 (95%CI: 1.07‐6.23) in male. However, the NPC incidence is much lower in female compared with male, might be due to very low smoking rate among female.

The NPC histological type in the endemic region is different from nonendemic area, nonkeratinizing carcinoma accounted for approximately 95% of NPC‐endemic regions and less than 65% in nonendemic regions.^44^, ^45^ And nonkeratinizing carcinoma is consistently associated with EBV infection,^46^ it seems that this cancer was more strongly related to EBV infection compared to smoking. In our study, about 94.37% (67/71) of NPC cases were nonkeratinizing carcinoma. We also found that EBV seropositivity was 85.92% (61/71) for VCA‐IgA (+) or EBNA1‐IgA (+) before NPC case detection and the aHR of EBV seropositivity was obviously higher than smoking.

Smoking has been proposed to interact with EBV through activating the virus to induce and promote NPC development.^28^ However, prospective evidence was lacking. Using stratification analyses, we observed the aHR for NPC was largely increased among the individuals who smoked and were EBV seropositive. Given the relatively small numbers of NPCs (n = 71) in each combination category, a real interaction between smoking and EBV could not be ruled out. These results were similar to the findings of Hsu et al in Taiwan, who found the highest risk in the subgroup for those who were EBV seropositive and heavy cigarette smokers. The lack of significant interaction might be due to a limited number of NPC cases.^42^ Larger, prospective studies are still needed to shed light on the interaction between EBV and smoking on NPC pathogenesis.

Considering EBV could be reactivated several years before NPC diagnosed, it is unreasonable to assess the relationship between smoking and EBV reactivation among NPC patients, even in the preclinical stage. An alternative way to test if smoking could induce EBV reactivation is to conduct the study in non‐NPC controls. Based on the NPC screening cohort with repeated testing for EBV serological screening markers, we evaluated the long‐term effects of smoking on EBV reactivation status. Whether at baseline, or the 3‐5 years of follow up, our results showed high consistency for the positive relationship between ever smoking and EBV antibodies seropositivity. Either current smokers or former smokers, the risks of EBV positivity were significantly higher compared with never smokers, with OR range from 1.30 to 2.00. By generalized estimating equation, similar results were also confirmed in the individuals who were tested more than three times. The results indicate that smoking has a long‐term effect on EBV reactivation, even after quitting smoking.

Although the mechanism for smoking reactivating latent EBV in B lymphocytes into lytic cycle is unknown, the inflammation and cell‐mediated immune reactions caused by cigarettes may be involved.^47^, ^48^ Once the virus in B lymphocytes is activated, they may enter into the circulation and nasopharynx. The switch is marked by the elevated EBV antibodies against viral antigens, such as VCA‐IgA, and EBNA1‐IgA. Furthermore, the proliferated B lymphocytes infected with EBV could also efficiently mediate the cell‐to‐cell contact mode for EBV infection into the epithelial cells.^49^ Under constant attacks from the virus, genetic instability increases and subsequently induces the epithelial cells into tumorigenesis.^50^ On the other hand, cigarette smoking can produce some DNA mutagens and damaging agents, which may drive cancer initiation in normal epithelial cells of the nasopharynx.^51^, ^52^

The main strength of this study is the prospective design, long‐term follow‐up to explore the association between smoking and NPC. Our results provide the prospective evidence for the etiological relationship between smoking and NPC incidence in endemic areas, and first prospectively suggested smoking might increase NPC risk by persistently activating EBV. Moreover, we analyze EBV reactivation responses to smoking with the longitudinal detection of two EBV antibodies (VCA‐IgA and EBNA1‐IgA). The consistent results for smoking and repeated EBV reactivation in different intervals further strengthen our conclusion. Since smoking and butyrates or nitrosamine intake is an oral‐nasopharyngeal process, the option of testing EBV DNA load in saliva or oral‐nasopharyngeal swabs should be added as markers of EBV reactivation and NPC presence 53, 54, 55, 56 in the future.

This study has some limitations. This cohort is based on a screening study, thus selection bias in the form of volunteer bias may exist. However, the prevalence of ever smoking among males (68.64%) and females (3.39%) in this cohort is consistent with the general population of southern China,^38^, ^42^ which indicates that the participants are representative of the source population for NPC cases in terms of smoking. Secondly, the information on smoking amount and smoking duration is not included in the questionnaire, which limits our further analysis for smoking indicators with the association of NPC risk. The third is that we just investigate smoking status at baseline and not to obtain the information at retesting EBV phase for the participants. The change of smoking habit may affect the association between smoking and NPC. Considering the change of smoking status may underestimate the NPC risk association with smoking,^42^ our results were then conservative.

## 5 CONCLUSION

In conclusion, our study reveals prospective evidence that smoking may increase the risk of NPC partly by repeatedly reactivating EBV. Considering the high prevalence of smoking, decreasing smoking rate might be an effective way to mitigate NPC incidence in endemic areas.

## AUTHOR CONTRIBUTIONS

T. Hu conducted questionnaire investigation, completed data analyses, and wrote the manuscript. C.‐Y. Lin conducted questionnaire investigation, collected important data during follow up, and gave advice on data analysis. S.‐H. Xie participated in data collection and managed the database. G.‐H. Chen conducted questionnaire investigation and blood sample collection. Y.‐Q. Lu, W. Ling, and Q.‐H. Huang engaged in recruitment of study population or acquisition of data. Q. Liu and S.‐M. Cao designed the study. Q. Liu provided support on statistics and S.‐M. Cao revised the manuscript for important intellectual content.

## CONFLICT OF INTEREST

All the authors declare no conflicts of interest in this work.
